# Fast Independent Component Analysis Algorithm-Based Diagnosis of L5 Nerve Root Compression and Changes of Brain Functional Areas Using 3D Functional Magnetic Resonance Imaging

**DOI:** 10.1155/2021/5063021

**Published:** 2021-07-22

**Authors:** Bofeng Zhao, Fuxia Yang, Lan Guan, Xinbei Li, Yuanming Hu, Chunlei Zhang, Yang Liu, Xiutao Li, Wucheng Wen, Hanqing Lyu

**Affiliations:** ^1^Department of Radiology, Shenzhen Traditional Chinese Medicine Hospital, The Fourth Clinical Medical College of Guangzhou University of Chinese Medicine, Shenzhen 518033, Guangdong, China; ^2^Department of Acupuncture and Moxibustion, Shenzhen Traditional Chinese Medicine Hospital, The Fourth Clinical Medical College of Guangzhou University of Chinese Medicine, Shenzhen 518033, Guangdong, China; ^3^Department of Clinical Laboratory, Shenzhen Traditional Chinese Medicine Hospital, The Fourth Clinical Medical College of Guangzhou University of Chinese Medicine, Shenzhen 518033, Guangdong, China

## Abstract

In this paper, the application of 3-dimensional (3D) functional magnetic resonance imaging (FMRI) in the diagnosis of the 5^th^ lumbar (L5) nerve root compression and brain functional areas in patients with lumbar disc herniation (LDH) was analyzed. The traditional fast independent component analysis (Fast ICA) algorithm was optimized based on the modified whitening matrix to establish a new type of Modified-Fast ICA (M-Fast ICA) algorithm that was compared with the introduced traditional Fast ICA and ICA. M-Fast ICA was applied to the 3D FMRI diffusion tensor imaging (DTI) evaluation of 65 patients with L5 nerve root pain due to LDH (group A) and 50 healthy volunteers (group B). The values of fractional anisotropy (FA) and apparent diffusion coefficient (ADC) in the lumbar nerve roots (L3, L4, L5, and the 1^st^ sacral vertebra (S1)) were recorded among subjects from the two groups. Besides, the score of edema degree in the lumbar nerve roots (L5 and S1) and activity of brain functional areas were also recorded among all subjects of the two groups. The results showed that the mean square error of M-Fast ICA was smaller than that of traditional Fast ICA and ICA, while its signal-to-noise ratio (SNR) was greater than that of Fast ICA and ICA (*P* < 0.05). The FA of L5 and S1 nerve roots in patients of group A was sharply lower than the values of group B, while the ADC of patients in group A was greater than that of the control group (*P* < 0.05). Besides, the score of edema in L5 and S1 nerve roots of patients in group A increased in contrast to group B (*P* < 0.05). The brain areas were activated after surgery including bilateral temporal lobe, left thalamus, splenium of corpus callosum, and right internal capsule. In conclusion, the 3D image denoising performance of M-Fast ICA optimized and constructed in this study was superior to that of the traditional Fast ICA and ICA. The FA of patients with L5 nerve root pain due to LDH decreased steeply, while the ADC increased dramatically. L5 nerve root pain caused by LDH resulted in changes in brain functional areas of the patients to inhibit the resting state default network activity, and the corresponding brain functional areas could be activated through treatment.

## 1. Introduction

LDH is a common and frequent-occurring disease in spine surgery, and low back pain and lumbocrural pain are the most common causes. Its clinical manifestations include low back pain, sciatica, and lower extremity radiation pain and weakness, and patients with severe symptoms suffer from incontinence of defecation and urination and abnormal sensation in the saddle area [1, 2]. Moreover, the main pathogenic factors of this disease include degenerative changes, annulus fibrosus disruption, or nerve root and cauda equina nerve stimulated and compressed by disc herniation in various parts of lumbar intervertebral disc (nucleus pulposus, annulus fibrosus, and cartilage plate) [3]. In addition, the incidence of L4-L5 and L5-S1 is the highest of patients with LDH, accounting for about 95% of the whole symptoms, while the incidence of multiple intervertebral disc herniation only occupies about 15%. LDH tends to emerge in young adults aged 20–40 years old (more males suffer from this disease than females), and it is often common in information technology (IT) practitioners, teachers, civil servants, drivers, and other long-term office workers [4, 5]. Excessive bending down should be avoided in life, and the back muscle should be exercised in order to improve lumbar muscle strength. Generally speaking, LDH cannot be completely cured, and most patients need mild conservative treatment to alleviate the disease. Therefore, it is very important to discuss the compression conditions of each lumbar vertebra in patients with LDH [6].

With the rapid development of imaging, MRI has been gradually applied in the diagnosis of LDH. By comparing with multiple indicators, it can clearly show the height, outline, annular tear, and high signal area of the intervertebral disc, with advantages of multidimensional imaging, high resolution, and high sensitivity. However, conventional MRI has a false positive rate and false negative rate in the diagnosis of elderly patients with lumbar nerve root pain, so it is necessary to adopt more excellent diagnostic tools [7,8]. Theoretically speaking, FMRI is designed to reflect the functional states of tissues and organs, and DTI, as an extension technique of conventional MRI, can visually display highly anisotropic nerve fibers [9]. On this basis, 3D MRI can process the cross-sectional images of any part or direction of one scan through electronic computers to form a 3D image, which can be further applied to diagnose the patient. ICA has been a new signal processing technology since the 1990s and mainly refers to the way to separate the source signals from the linear mixed signals of multiple source signals, which is featured with rapid convergence. However, it is easy to be interfered with by the SNR of data when processing FMRI data, which affects the results of analysis [10, 11]. Therefore, this study intended to optimize Fast ICA to explore its value in the MRI diagnosis of LDH.

To sum up, ICA is a traditional method for FMRI denoising, but it has some defects. On this basis, the traditional Fast ICA was optimized through the modified whitening matrix to construct the M-Fast ICA, so as to apply to the DTI evaluation of 65 patients with L5 nerve root pain due to LDH (group A) and 50 healthy volunteers (group B). Besides, the traditional Fast ICA and ICA were compared with M-Fast ICA. The FA and ADC of L3, L4, L5, and S1 lumbar nerve roots and brain activation areas after surgery in patients from the two groups were compared to comprehensively evaluate the application of FMRI in the diagnosis of L5 nerve root compression and brain functional areas in patients with LDH.

## 2. Materials and Methods

### 2.1. Sample Selection

In this study, 65 patients with L5 nerve root pain due to LDH were selected as group A, who were admitted to the hospital from January 1, 2019, to July 15, 2020; and 50 healthy volunteers were selected as group B, who underwent physical examination during the same period. During the surgery, the edema degree of the diseased nerve roots was evaluated based on the color of nerve roots (1 point for yellow-white, 2 points for pink, and 2 points for purplish red) and the thickness (0 points for no obvious thickening and 1 point for thickening). In addition, the higher the score, the greater the edema. This study had been approved by the Medical Ethics Committee of the hospital. Moreover, the subjects and their family members had known about this study and signed informed consent and failed examination consent.

The criteria for inclusion were defined to include the subjects who were older than 18 years old, were right-handed, had clear consciousness, could cooperate with the examination, were diagnosed with LDH accompanied by root pain, and suffered from LDH of the unilateral lower extremity.

The criteria for exclusion were defined to include the subjects who were pregnant, suffered from cardiovascular diseases, had taken relevant drugs, had mental diseases, and interrupted the examination.

### 2.2. Magnetic Resonance Imaging Scanning

MR Prisma 3.0 magnetic resonance machine produced by Siemens, Germany, was adopted to scan all subjects. Subjects were placed in the supine position with quiet breathing. Standard Siemens spinal coils were placed in the subject's scanning sequence and scanned based on the location of LDH. Conventional MRI scan parameters were shown as follows: the repeat time was 4,500 ms, echo time was 115 ms, field of view was 250 × 250 mm, matrix was 251 × 325, the thickness of a layer was 3.5 mm, and the number of layers was 10. The scan parameters of DTI included repeat time of 7,500 ms, echo time of 82 ms, view field of 310 × 150 mm, matrix of 108 × 308, thickness of 3.5 mm, layer number of 40, and scanning time of 20 minutes. The obtained image sent to the workstation was completed after the scanning, and the Neuro Space was employed to select the region of interest (near the lumbar intervertebral foramen) to measure the FA and ADC. What is more, the activation rate of each brain area was recorded (it indicated that the low-frequency fluctuation amplitude was active brain area with statistical significance when the voxel value in the magnetic resonance image was equaled to or more than 2.262).

### 2.3. Magnetic Resonance Imaging Denoising Algorithm Based on Fast Independent Component Analysis Algorithm

Fast ICA was a fixed point recursive algorithm proposed by Hyvarinen et al. from the University of Helsinki, Finland. With its fast convergence speed and good separation effect, Fast ICA was widely applied in signal processing and could well estimate the mutually statistically independent original signals mixed by unknown factors from the observed signals. This algorithm firstly centralized the observed signals so that the mean vectors of the observed signals were all 0, and then, the centralized observed signals were whitened. It could be expressed as follows:

(1) $$\begin{array}{c} F=W_{N}\left(S-\bar{S}\right), \end{array}$$

where *S* stood for an observed signal, $\bar{S}$ expressed the mean vector of an observed signal, *W*_*N*_ represented a whitening matrix, and *f* stood for a whitened signal. Then, the matrix *N* was initially separated so that ‖*N*‖=1. The matrix should be updated, and the iterative processing was for the separated matrix by Newton iteration method to obtain *N*_1_ that was orthogonalized. Thus, the matrix *N* was shown as the following equation:

(2) $$\begin{array}{c} N={\left(N_{1}N_{1}^{T}\right)}^{-\left(1/2\right)}N_{1}, \end{array}$$

where *T* represented the orthogonalization factor. Finally, the convergence of the separated matrix *N* was judged. If the convergence state was reached, the optimal estimation value of the source signal at this time could be calculated as follows:

(3) $$\begin{array}{c} \overset{⟶}{U}=NS, \end{array}$$

where *U* stood for a source signal. If the separation matrix *N* did not converge, the return iteration continued until it converged. Considering that the traditional Fast ICA did not exclude the interference of image noise to the signal during whitening, the whitening processing was optimized and the whitening matrix was formed by the combination of eigenvalues of the noise subspace and the eigenvalues of the signal subspace. Firstly, the autocorrelation matrix of the observed matrix was obtained through the following equation:

(4) $$\begin{array}{c} R_{ss}=G\left[SS^{T}\right], \end{array}$$

where *R*_*ss*_, *T*, and *G*[·] expressed the autocorrelation matrix, the orthogonalization factor, and the autocorrelation function, respectively. Then, the eigenvalues were discomposed, as shown in the following:

(5) $$\begin{array}{c} R_{ss}=V_{s}\exists V_{S}^{H}, \end{array}$$

where ∃, *V*, and *H* represented the eigenvalue corresponding to signal subspace, the eigenvalue vector corresponding to signal subspace, and the signal factor of the matrix, respectively. Besides, ∃=diag(*λ*_1_, *λ*_2_,…, *λ*_*n*_) and *V*_*S*_^*H*^=[*V*_*i*_/*V*_*n*−*i*_]^*H*^. Thus, the whitening matrix was formed by the eigenvalues and eigenvalue vectors, which was expressed in the following equation:

(6) $$\begin{array}{c} N=\exists_{i}^{-\left(1/2\right)}V_{i}^{H}. \end{array}$$

Then, the main eigenvalue was modified to obtain the following:

(7) $$\begin{array}{c} \overset{↔}{\exists_{i}}=\exists_{i}-{\bar{\Delta }}^{2}\sigma_{i}, \end{array}$$

where $\overset{↔}{\exists_{i}}$ stood for the main eigenvalue after modification, ${\bar{\Delta }}^{2}$ expressed the weight matrix corresponding to the average eigenvalue of noise, and *σ*_*i*_ represented the weight matrix corresponding to the eigenvalues of the signal subspace. What is more, ${\bar{\Delta }}^{2}=\sum_{i+1}^{n}\left(\lambda_{i+1}/\left(n-i\right)\right)$ and *σ*_*i*_=diag(*σ*_1_, *σ*_2_,…, *σ*_*n*_). The new whitening matrix could be calculated as follows:

(8) $$\begin{array}{c} N={\overset{↔}{\exists_{i}}}^{-\left(1/2\right)}V. \end{array}$$

The above was the M-Fast ICA optimized on the basis of the modified whitening matrix, which fully considered the impact of noise and helped to separate the signal with low signal noise.

### 2.4. Evaluation Indicators of Image Enhancement Performance

The traditional Fast ICA [12] and ICA [13] were introduced to compare with M-Fast ICA constructed in this study. The root mean square error (RMSE) and SNR were regarded as evaluation indicators.

RMSE referred to the square root of the variance between the original signal and the denoised signal, which can be expressed as follows:

(9) $$\begin{array}{c} \text{RMSE}={\left\{\frac{{\left[f\left(n\right)-f{\left(n\right)}^{*}\right]}^{2}}{n}\right\}}^{1/2}, \end{array}$$

where *f*(*n*) and *f*(*n*)^*∗*^ stood for the original signal and the denoised signal, respectively.

SNR was a traditional method for detecting noise measurement in signals, which can be calculated as the following:

(10) $$\begin{array}{c} \text{SNR}=10\;\log\;10\left(\frac{P_{s}}{P_{z}}\right), \end{array}$$

where *P*_*s*_ and *P* represented the power of the original signal and the power of noise, respectively. In addition, *P*_*s*_={[∑*f*^2^(*n*)]/*n*} and *P*_*z*_=RMSE^2^.

### 2.5. Statistical Methods

SPSS19.0 version statistical software was adopted to analyze the data processing in the study, measurement data were expressed as mean ± standard deviation, and enumeration data was represented by percentage (%). The SNR and RMSE of Fast ICA, ICA, and M-Fast ICA were pairwise compared through the one-way variance analysis. The independent *t*-test was applied to compare the FA and ADC of the lumbar nerve roots (L3, L4, L5, and S1) with the edema degree score of the lumbar nerve roots (L5 and S1) of the subjects in the two groups. *P* < 0.05 meant the difference was statistically significant.

## 3. Results

### 3.1. Comparison of Basic Information of the Subjects in the Two Groups

Figure 1 shows the comparison of basic information of the subjects in the two groups. It indicates that the age of the subjects in group A was 50.17 ± 8.83 years old, the height was 160.21 ± 12.33 cm, the weight was 58.28 ± 7.82 kg, the male proportion was 56.08%, and the female proportion was 43.92%. Besides, the age, height, weight, male proportion, and female proportion of the subjects in group B were 51.62 ± 8.91 years old, 162.13 ± 10.56 cm, 59.41 ± 7.07 kg, 53.81%, and 46.19%, respectively. There were no great differences in the age, height, weight, male proportion, and female proportion of the subjects from groups A and B (*P* > 0.05).

### 3.2. Comparison of the Root Mean Square Error and Signal-to-Noise Ratio of the Three Algorithms

Figure 2 indicates the comparison of RMSE and SNR of the three algorithms. It reveals that the values of RMSE in the ICA, Fast ICA, and M-Fast ICA were 6.38 ± 0.52, 6.25 ± 0.72, and 4.91 ± 0.38, respectively; and the values of SNR in the ICA, Fast ICA, and M-Fast ICA were 71.42 ± 5.49 dB, 72.37 ± 5.18 dB, and 86.36 ± 6.77 dB, respectively. Therefore, the RMSE of M-Fast ICA was obviously higher than the values of ICA and Fast ICA, showing a statistical substantial difference (*P* < 0.05). However, the SNR of M-Fast ICA increased dramatically in contrast to ICA and Fast ICA, with a statistical great difference (*P* < 0.05).

Figure 3 expresses the MRI image reconstruction results of the lumbar spine by the three algorithms. Figure 3 shows the original ultrasound image of one patient, with a blurred lumbar spine and a lot of noise. The image resolution of M-Fast ICA was higher markedly than that of ICA and Fast ICA after denoising, and the noise reduction was obvious, so M-Fast ICA could fully meet the requirements of clinical imaging diagnosis.

### 3.3. Comparison of the Fractional Anisotropy of the 3^rd^, 4^th^, and 5^th^ Lumbar and the 1^st^ Sacral Vertebra Nerve Roots in the Subjects from Both Groups

Figure 4 shows the comparison of FA of L3 and L4 lumbar nerve roots among the subjects in the two groups. It was known that the FA of L3 and L4 lumbar nerve roots were 314.24 ± 17.71 and 308.41 ± 17.55 in patients from group A, respectively. Besides, the FA of L3 lumbar nerve root was 319.41 ± 30.31 and the FA of L4 lumbar nerve root was 315.76 ± 27.45 in the subjects from group B. The values of FA in L3 and L4 lumbar nerve roots of patients from group A were not statistically considerable in contrast to group B (*P* > 0.05).

Figure 5 indicates the comparison of FA in the L5 and S1 lumbar nerve roots among the subjects from the two groups. The FA of L5 lumbar nerve root was 250.58 ± 16.62 and its S1 lumbar nerve root was 239.64 ± 18.85 in patients of group A; and the values of FA in L5 and S1 lumbar nerve roots were 331.71 ± 18.93 and 316.46 ± 28.82, respectively. Among them, the values of FA in the L5 and S1 lumbar nerve roots were lower sharply in patients of group A than those of group B, and the difference was statistically remarkable (*P* < 0.05).

### 3.4. Comparison of the Apparent Diffusion Coefficient of the 3^rd^, 4^th^, and 5^th^ Lumbar and the 1^st^ Sacral Vertebra Nerve Roots in the Subjects from Both Groups

In Figure 6, there are comparisons of the ADC of L3, L4, L5, and S1 lumbar nerve roots among the subjects in the two groups. It was observed that the values of ADC in the L3, L4, L5, and S1 lumbar nerve roots were 0.64 ± 0.025 × 10^3^ s/mm^2^, 0.52 ± 0.016 × 10^3^ s/mm^2^, 0.86 ± 0.024 × 10^3^ s/mm^2^, and 0.79 ± 0.033 × 10^3^ s/mm^2^ in the patients from group A, respectively. What is more, the values of ADC in the S1, L3, L4, and L5 lumbar nerve roots were 0.58 ± 0.011 × 10^3^ s/mm^2^, 0.71 ± 0.018 × 10^3^ s/mm^2^, 0.54 ± 0.021 × 10^3^ s/mm^2^, and 0.51 ± 0.016 × 10^3^ s/mm^2^ in the subjects from group B, respectively. The ADC of the L3 and L4 lumbar nerve roots in the subjects from group A was not statistically substantial compared with that of group B (*P* > 0.05). However, ADC of the L5 and S1 lumbar nerve roots in the subjects from group A increased enormously in contrast to group B, and there was a statistically obvious difference (*P* < 0.05).

### 3.5. The Edema Scoring of the 3^rd^, 4^th^, and 5^th^ Lumbar and the 1^st^ Sacral Vertebra Nerve Roots in the Subjects from the Two Groups

There was a comparison of edema scoring of the L5 and S1 lumbar nerve roots among the subjects in the two groups, as shown in Figure 7. It revealed that the edema scores of the L5 and S1 lumbar nerve roots were 5.62 ± 1.43 and 4.07 ± 1.13 in the patients of group A, respectively. The edema scores of the L5 and S1 lumbar nerve roots were 1.62 ± 0.33 and 1.25 ± 0.24 in the patients of group B, respectively. Among them, the edema scores of the L5 and S1 lumbar nerve roots were higher hugely in the subjects of group A than those of group B, indicating a statistically great difference (*P* < 0.05).

### 3.6. Brain Areas with Higher Activation Rates in the Patients of Group A after Surgery

Figure 8 shows the brain regions after surgery with a higher rate of activation in all patients of group A. It indicates that the activation rates of the left temporal lobe, right temporal lobe, left thalamus, splenium of corpus callosum, and right internal capsule were 100%, 100%, 100%, 68.31%, and 87.43%, respectively.

## 4. Discussion

LDH is a very common medical lesion, with about 80% of people experiencing low back pain in their lifetime. Herniated lumbar disc can lead to lumbar nerve root compression, so as to let patients suffer from sciatica, and the area with the highest incidence is the gap between the L4 and L5 lumbar roots [14]. The 3D FMRI is a typical method for the clinical diagnosis of LDH. Due to various objective factors that cause the original FMRI image quality, the traditional Fast ICA was optimized based on the modified whitening matrix to establish the M-Fast ICA, and the traditional Fast ICA and ICA were introduced for simulation denoising comparison with M-Fast ICA. The results showed that the RMSE of M-Fast ICA was greater markedly than that of ICA and Fast ICA, indicating that the difference was statistically obvious (*P* < 0.05), while the SNR of M-Fast ICA was smaller extremely than that of ICA and Fast ICA, suggesting that there was a statistically huge difference (*P* < 0.05). It was similar to the research results of Ariyasu et al. [15], showing that the denoising effect of M-Fast ICA constructed in this study with good generalization was far better than that of Fast ICA and ICA for FMRI images. Under the reconstruction results of lumbar neurological MRI images by the three algorithms, the image definition after denoising by M-Fast ICA was higher dramatically than that of ICA and Fast ICA, and the noise reduced sharply. In addition, it was consistent with the above quantitative data results and also demonstrated the superiority of M-Fast ICA [16].

M-Fast ICA was applied to evaluate the DTI of 65 patients with L5 nerve root pain caused by LDH (group A) and 50 healthy volunteers (group B). The results suggested that the FA of L3 and L4 lumbar nerve roots in the subjects of group A were not statistically extreme compared with that of group B (*P* > 0.05), which was similar to the research results of Wang et al. [17], indicating that patients with L5 nerve root pain caused by LDH had no lesion changes in L3 and L4 lumbar nerve roots, which were not different from healthy volunteers. The FA of L5 and S1 lumbar nerve roots was lower steeply in the subjects of group A than that of group B, and the difference has statistical significance (*P* < 0.05), which was different from the results of Wu et al. [18]. It might be associated with histopathological changes in nerve roots generated from the nerve root compressed by herniated disc, and DTI images presented the disorder and narrow of nerve fibers and the decline of FA. The ADC of L3 and L4 lumbar nerve roots in the subjects from group A was not statistically substantial compared to that of group B (*P* > 0.05), but its ADC of L5 and S1 lumbar nerve roots was higher greatly than that of group B (*P* < 0.05). Chronic compression of the same lumbar nerve roots would lead to changes of edema and hyperemia in the nerves, and their continuous development would even reduce blood flow to the blood vessels, resulting in nerve root ischemia; thus, the ADC increased. The edema score of L5 and S1 lumbar nerve roots in the patients from group A was obviously higher than that of group B, and the difference was statistically remarkable (*P* < 0.05), indicating that there were pathological tissue changes and the increasing edema degree of the nerve roots in patients with LDH [19]. The activation rates of the right temporal lobe, left temporal lobe, left thalamus, right internal capsule, and splenium of corpus callosum were 100%, 100%, 100%, 87.43%, and 68.31%, respectively, in the patients of group A. Therefore, it revealed that the L5 nerve root pain result caused by LDH led to the changes in the brain functional area to restrain the resting state of the default network activity, which could be activating the corresponding brain regions through treatment.

## 5. Conclusion

This study optimized the traditional Fast ICA based on the modified whitening matrix to construct the M-Fast ICA that was compared with the introduced traditional Fast ICA and ICA. Moreover, M-Fast ICA was adopted to the 3D DTI evaluation of 65 patients with L5 nerve root pain caused by LDH and 50 healthy volunteers. It was found that the image denoising performance of M-Fast ICA constructed in this study was better than the traditional Fast ICA and ICA. The FA of patients with L5 nerve root pain caused by LDH dropped sharply but its ADC rose obviously. Changes in the functional areas of the patient's brain were affected by L5 nerve root pain caused by LDH to inhibit the resting state default network activity, and the corresponding brain functional areas could be activated by the treatment. However, the number of lumbar disc herniation patients with L5 nerve root pain was relatively small in this study and from a single source, which was less supportive of the results. Therefore, the sample size of patients should be increased in the future to further explore the application value of Fast ICA. In summary, the results of this study provided a theoretical basis for the clinical diagnosis of nerve roots in patients with lumbar disc herniation.

## Figures and Tables

**Figure 1:** Comparison of basic information of the subjects in both groups. (a) Comparison of the age, height, and weight of the subjects in groups A and B; (b) comparison of the male and female proportion of the subjects in the two groups.

**Figure 2:** (a, b) Comparison of RMSE and SNR of the three algorithms. ^*∗*^There was a statistical difference in contrast to M-Fast ICA (*P* < 0.05).

**Figure 3:** MRI image reconstruction results of lumbar nerves by the three algorithms. (a) Original MRI image of a male patient; (b) image denoised by ICA; (c) image denoised by Fast ICA; and (d) image denoised by M-Fast ICA.

**Figure 4:** Comparison of FA of L3 and L4 lumbar nerve roots among the subjects in both groups.

**Figure 5:** Comparison of FA of L5 and S1 lumbar nerve roots among the subjects in both groups. ^*∗*^There was a statistical difference in contrast to group B (*P* < 0.05).

**Figure 6:** Comparison on ADC of the L3, L4, L5, and S1 lumbar nerve roots among the subjects in the two groups. ^*∗*^The difference was statistically significant in contrast to group B (*P* < 0.05).

**Figure 7:** Comparison of the edema scores of the L5 and S1 lumbar nerve roots among the subjects in both groups. ^*∗*^The difference was statistically obvious in contrast to group B (*P* < 0.05).

**Figure 8:** Brain regions with a higher activation rate in the patients of group A after surgery. 1, 2, 3, 4, and 5 stand for the activation rates of the left temporal lobe, right temporal lobe, left thalamus, splenium of corpus callosum, and right internal capsule in sequence.

## Data Availability

No data were used to support this study.
